This article has been retracted.

# The impact of horse purslane (*Trianthema portulacastrum* L.) infestation on soybean [*Glycine max* (L.) Merrill] productivity in northern irrigated plains of Pakistan

**DOI:** 10.1371/journal.pone.0257083

**Published:** 2021-09-20

**Authors:** Khuram Mubeen, Muhammad Shehzad, Naeem Sarwar, Haseeb ur Rehman, Tauqeer Ahmad Yasir, Allah Wasaya, Matlob Ahmad, Mubshar Hussain, Muhammad Bilal Abbas, Muhammad Waqas Yonas, Shahid Farooq, Tahani Awad Alahmadi

**Affiliations:** 1 Department of Agronomy, MNS University of Agriculture, Multan, Pakistan; 2 Department of Agronomy, The University of Poonch, Rawalakot, AJK, Pakistan; 3 Department of Agronomy, Bahauddin Zakaria University, Multan, Pakistan; 4 College of Agriculture, Bahauddin Zakaria University, Layyah, Pakistan; 5 Department of Agricultural Engineering and Technology, Ghazi University, Dera Ghazi Khan, Pakistan; 6 Department of Plant Protection, Faculty of Agriculture, Harran University, Şanlıurfa, Turkey; 7 Department of Pediatrics, College of Medicine, King Saud University, [Medical City], King Khalid University Hospital, Riyadh, Saudi Arabia; Mendel University of Agriculture and Forestry: Mendelova univerzita v Brne, CZECH REPUBLIC

## Abstract

Horse purslane (*Trianthema portulacstrum* L.) is an important weed of soybean crop capable of causing significant yield reduction. Therefore, this study assessed the impact of horse purslane and other weeds’ infestation on the productivity of soybean. Ten treatments, i.e., weed-free throughout the growing season, horse purslane-free till 20, 40 and 60 days after emergence (DAE), all weeds-free till 20, 40 and 60 DAE, weedy-check (excluding horse purslane), weedy-check (horse purslane alone) and weedy-check (all weeds) were included in the study. Data relating to density and dry weight of recorded weed species, and yield and related traits of soybean were recorded. Overall, infestation percentage of horse purslane was 33.10 and 51%, whereas dry weight was 12 and 44 g m^-2^ during 1^st^ and 2^nd^ year, respectively. The highest dry weight of all weed species was recorded at 45 DAE in weedy-check all weeds treatment during both years. The lowest relative density and frequency of horse purslane were recorded in the treatment where it was controlled until 20 DAE during 2018 at 30 DAE, whereas the same treatment recoded the lowest density of horse purslane at 45 DAE during 2019. The relative frequency of horse purslane was non-significant for weedy-check horse purslane and weedy-check all weeds treatments during 2018, whereas former treatment had higher relative frequency of horse purslane in weedy-check all weeds than the later during 2019. Yield and related traits significantly differed among different treatments used in the study. The treatment all weeds controlled until 40 DAE recorded higher number of pods per plant, 1000-seed weight and seed yield during both years. The yield reduction in weedy-check treatments was; weedy-check all weeds > weedy-check all weeds except horse purslane > weedy-check horse purslane only. It is concluded that horse purslane was not the sole weed interfering soybean fields and weed flora consisted of false amaranth [*Digera muricata* (L.) Mart.] and purple nut sedge (*Cyperus rotundus* L.). Hence, if the soybean fields in northern irrigated plains of Pakistan are infested with horse purslane or heavily infested with horse purslane or other weeds, these should be controlled in initial 40 DAE to improve soybean productivity.

## Introduction

Soybean [*Glycine max* (L.) Merrill], a member of the Fabaceae family, is one of the most valuable oilseed crops, mainly grown for edible seed around the world. It is an annual plant, generally grows to a height of 20–180 cm and bears white or lilac flowers and pods [1]. Soybean, like other legumes, has the ability to fix nitrogen from the air; thus, useful for crop rotation [2]. It is the most economical source of edible oil (18–22%) and rich in protein contents (~40%) [3]. It is the only source of vegetable oil that contains complete protein [4].

Soybean can provide two fold more protein than any other vegetable or grain crop [5]. During 2019, it was planted on 122.44 million hectares globally with 336.59 million metric tons (MMT) of seed production. Brazil is the largest producer of soybean with 126.00 MMT seed production annually followed by the USA (96.67 MMT) and Argentina (49.00 MMT). The global soybean production was estimated to reach 369.74 MMT during 2020 [6]. Pakistan is an agricultural country, where most of the population is reliant on agriculture and its products. However, the country is spending huge amount of money on edible oil import. Pakistan imports soybean for livestock feed industry and ~2.0 MMT soybean was imported during 2019 [7]. Weed infestation is a yield limiting factor in soybean production, mainly due to its plantation in summer season, which is followed by monsoon rains and subsequent weeds’ infestation [8]. Several factors are responsible for the lower area under cultivation of the crop are, lack of marketing of produce and its byproducts, and absence of adequate skills, knowledge and production technology. Moreover, lack of high yielding, climate and pest resistant varieties is the other major bottleneck in the cultivation and adaptation of soybean in Pakistan [3].

Weed interference is a complex and persistent limitation in soybean production in many states of the world. Weed infestation poses negative impacts on soybean growth and development [9–13]. Heavy weed infestation in soybean interferes with the timelines and efficiency of harvests. Severe yield losses are observed in soybean if weeds are left unaddressed [14]. Grain yield reduction due to weed infestation in soybean in India varies from 27% to 77%, depending on weed species, soil type, cropping season and severity of weed infestation [15]. Like other major crops, prolonged weed infestation in soybean can result in significant yield and quality losses. Thus, early weed control is necessary to achieve higher yield and improve productivity and economic returns of soybean [16].

Horse purslane (*Trianthema portulacastrum* L.), a member of the Aizoaceae family has emerged as a significant threat to the sustainability of the soybean production systems globally. It is rapidly spreading and regarded as a noxious weed in Punjab province of Pakistan. The infestation of horse purslane alone resulted in 10.81% higher yield reduction than infestation of all weeds in southern Punjab, Pakistan [17]. Horse purslane is a prostrate, branched, fast-growing and succulent annual plant with green leaves. It produces small white flowers and has a high fecundity rate. Horse purslane is native to South Africa, but widely distributed in India, Sri Lanka, West Asia and Pakistan [18]. It adversely effects the growth of crop plants globally [19]. Due to higher branching character and prostrate growth nature, it quickly covers the ground and forms a green carpet [20]. Compared with other weeds, horse purslane is more dangerous in the same crop field. It has the potential to reduce soybean stand by 60% and grain yield by 34% [17]. However, the documented information on the interference of horse purslane relative to other weeds in soybean fields in northern irrigated plains of Pakistan is scarce. This experiment was conducted in the soybean field in northern irrigated plains to compare the interference of horse purslane relative to other weeds and assess their effects on productivity of soybean.

## Materials and methods

### Experimental site

The experiments were conducted at research area of Muhammad Nawaz Shareef University of Agriculture, Multan, Pakistan. Experiments were conducted for two consecutive cropping years (2018 and 2019) in the same field. The region is irrigated with arid climate (30^o^ 12’ N, 71^o^ 28’ E and altitude 123 m) [21]. The study area receives average annual rainfall of 175 mm per year with an average annual temperature of 25.6°C [22]. The climatic conditions of the experimental site are presented in Figs 1 and 2. Soil of the experimental site is clay-loam with low organic matter content. Soybean seeds were manually sown keeping seed rate of 98 kg ha^-1^, plant-to-plant distance of 15 cm and 30 cm row-to-row spacing. Individual plot dimension was 1.5 m × 3.5 m, plot-to-plot space of 0.33 m and replications were separated by 1 m space. Nitrogen, phosphorus and potassium were used at 25, 50 and 50 kg ha^-1^ at sowing time and 15 kg ha^-1^ supplemental nitrogen was applied at flowering. Canal and tube well water was used for irrigation at 20 days interval. Total three irrigations were applied to the crop. Agronomic practices were retained same for all the treatments.

**Fig 1:** Climatic data of the experimental site during soybean growing season of 2018.

**Fig 2:** Climatic data of the experimental site during soybean growing season of 2019.

### Experimental design and treatments

The experiment comprised of ten treatments, i.e., weeds-free (whole season), horse purslane-free till 20, 40 and 60 days after emergence (DAE), all weeds-free till 20, 40 and 60 DAE, all weeds-free till 40 and 60 DAE, weedy-check (all weeds except horse purslane), weedy-check (horse purslane only) and weedy-check (all weeds). Experiments were arranged according to randomized complete block design with three replications. The crop was sown during the 1^st^ week of August in both years and cultivar ‘Faisal soybean’ obtained from Ayub Agriculture Research Institute, Faisalabad (Punjab, Pakistan) was used as experimental material. The seeds were inoculated with *Rhizobium phaseoli* before planting during both years. The inoculum was obtained from Department of Soil Bacteriology, Ayub Agriculture Research Institute, Faisalabad (Punjab, Pakistan).

### Observations

Data relating to weeds’ infestation percentage, dry weight, frequency percentage, relative frequency, relative weed density and yield-related parameters of soybean (number of pods plant^-1^, 1000-seed weight and seed yield) were recorded. Weed-related data were recorded by using quadrate of 1 m^-2^ at 15 days interval. All weed plants inside the quadrate were removed manually to record density and dried in an oven for 48 hours at 70°C for recording dry weight m^-2^. Density is the measure of the number of plants of a species in a given area (e.g. square meter or hectare). Frequency percentage was determined by using the method of Kilewa and Rashid [23]. Relative density, relative frequency and frequency percentage were determined by following Yakubu et al. [24] and Tauseef et al. [25].


$$Frequency\;\%=\frac{\mathrm{Number}\;\mathrm{of}\;\mathrm{sampling}\;\mathrm{unit}\;\mathrm{having}\;\mathrm{target}\;\mathrm{species}}{\mathrm{Total}\;\mathrm{number}\;\mathrm{of}\;\mathrm{sampling}\;\mathrm{unit}}\times 100$$

$$Relative\;frequency\;\%=\frac{\mathrm{Frequency}\;\mathrm{of}\;\mathrm{target}\;\mathrm{species}}{\mathrm{Sum}\;\mathrm{frequences}\;\mathrm{of}\;\mathrm{all}\;\mathrm{species}}\times 100$$

$$Relative\;density\;\%=\frac{\mathrm{Total}\;\mathrm{number}\;\mathrm{of}\;\mathrm{individuals}\;\mathrm{of}\;a\;\mathrm{particular}\;\mathrm{species}}{\mathrm{Total}\;\mathrm{number}\;\mathrm{of}\;\mathrm{individuals}\;\mathrm{of}\;\mathrm{all}\;\mathrm{weed}\;\mathrm{species}}\times 100$$

Plant height, 1000-grain weight and grain yield of soybean were recorded at maturity. Quadrate sampling method was used to assess number of pods per plant. Pods were manually detached from the plants and counted. After removing husk, seeds were taken-off from the pods and counted. Three random samples of 1000 grains from each treatment were weighed and averaged to record 1000-grain weight. The number of plants in 1 m^2^ were harvested and total grains present on the plants were weighed to record seed yield.

### Statistical analysis

The collected data on all attributes were tested for normality using Shapiro-Wilk normality test and data having non-normal distribution were normalized by Arcsine transformation technique. The differences among years were tested by paired t test, which indicated significant differences among years. Therefore, data of both years were analyzed, presented and interpreted separately. One-way analysis of variance (ANOVA) was used to test the significance in the data [26]. Tukey’s honestly significant difference test at 5% probability was used to separate the means where ANOVA indicated significant differences. All statistical computation were executed on SPSS statistical software version 20.

## Results and discussion

False amaranth [*Digera muricata* (L.) Mart.] recorded the highest infestation (64 and 48% during 2018 and 2019, respectively) in weedy-check all weeds treatment. Interestingly, horse purslane (*Trianthema portulacstrum* L.) recorded the highest dry weight in weedy-check all weeds treatment at 45 DAE during both years of the study (Fig 3).

**Fig 3:** Weed density (a) and dry biomass (b) in weedy-check all weeds treatment at 45 DAE in soybean during 2018 and 2019.

Weed flora consisted of horse purslane, false amaranth and purple nut sedge (*Cyperus rotundus* L.) during both years. The density of horse purslane was 12 plants m^-2^ during 1^st^ year; however, increased to 33 plants m^-2^ during 2^nd^ year. The increase in density during 2^nd^ year (by 21 plants m^-2^) is quite understandable and can be attributed to little seed dormancy and high seed dispersal in field at the end of first year because horse purslane can produce 33000 seeds per plant under favorable environmental conditions [27]. Moreover, higher rainfall during 2^nd^ year might have created a favorable micro soil and aerial environment, which stimulated the seed germination of horse purslane. Higher density of false amaranth than all other weed species during both years could be a reflection of its historic enriched soil seed bank. Although horse purslane had higher density than purple nut sedge during 2019, it had less density than false amaranth during both years. Horse purslane is more damaging at early stage when soybean canopy is not fully developed. It is strong competitor due to rapid growth, profuse branching and spreading growth habit, which help the weed to quickly cover the soil and form a green carpet that could reduce dry biomass of other weed species [28]. It could answer that why horse purslane had higher dry mass despite less density during 2018. In contrast, lower dry weight amid higher density could be explained by interplant competition for resources in horse purslane. The lower number of plants probably found more resources; thus, partitioned more assimilates, whereas higher density resulted in lower assimilate portioning.

Purple nut sedge was the most abundant weed after false amaranth during first year. However, density of purple nut sedge reduced in second year probably due to the difference in rainfall during both years. Higher infestation of horse purslane during second year could also be a likely reason. False amaranth infestation was also reduced during second year compared to first year and the differences were significant among years. It can again be associated with an increase in the infestation of horse purslane due to seed dispersal over time and area. Seed dispersal probably affected neighboring weed seeds and seedlings. The decline in dry weight of false amaranth and purple nut sedge could be due to strong competitive and allelopathic nature of horse purslane. Reduction in infestation percentage and dry biomass of false amaranth and purple nut sedge correlates with increased infestation and dry biomass of horse purslane. It can be attributed to higher seed production and ability to complete more than one life cycle in the same growing seasons with almost no seed dormancy constraint of horse purslane. All these traits collectively allowed horse purslane to produce higher biomass than other weed species [29].

The highest relative density of horse purslane was observed at 30 and 45 DAE in weedy-check horse purslane only treatment during both years (Fig 4). During 2019, higher rainfall stimulated germination of horse purslane, subsequent seedling emergence and better establishment in weedy-check horse purslane only treatment. The soybean plots where horse purslane was not allowed to grow until 20 DAE recorded the lowest relative density of horse purslane at 45 DAE (18.28 and 17.49% 1^st^ and 2^nd^ year, respectively). A slight increase in relative density of horse purslane was recorded at 45 DAE than 30 DAE as horse purslane was approaching its climax vegetative growth during this period.

**Fig 4:** Relative density of horse purslane in soybean field at 30 (a) and 45 (b) days after emergence. T_2_: Horse purslane-free till 20 DAE, T_5_: All weeds-free till 20 DAE, T_9_: Weedy check horse purslane only, T_10_: Weedy-check all weeds.

Relative frequency was recorded at different intervals to determine the specific period of dominance of each weed. Relative frequency indicates the degree of dominance of certain weed over other weeds present in the field at a certain period of time. The data presented in the Fig 5 indicated that the highest relative frequency was recorded at 30 DAE during both years.

**Fig 5:** Relative frequency of horse purslane at 30 (a) and 45 (b) days after emergence in soybean field. T_2_: Horse purslane-free till 20 DAE, T_5_: All weeds-free till 20 DAE, T_9_: Weedy check horse purslane only, T_10_: Weedy-check all weeds.

The highest relative frequency (RF) of horse purslane was recorded in weedy-check horse purslane only treatment, whereas in all weeds-free treatment until 20 DAE recorded the lowest RF at 30 DAE during 2018. However, during 2019, horse purslane-free treatment until 20 DAE recorded the lowest RF. Moreover, at 45 DAE, minimum RF was observed in the plots where horse purslane was controlled until 20 DAE during both years. At 45 DAE, the highest RF of horse purslane might be attributed to highly favorable environmental and soil conditions. The lowest RF of horse purslane was recorded at 30 DAE in all weeds-free treatment until 20 DAE.

The frequency of horse purslane at 30 DAE did not differ among weedy-check horse purslane only and weedy-check all weeds treatments during 2018 (Fig 6). However, lesser frequency was noted in weedy-check all weeds than weedy-check horse purslane alone treatment during 2019 at 30 DAE. This variation over years could be attributed to lesser rainfall during 2018. However, horse purslane and all weeds-free soybean plots until 20 DAE recorded higher frequency percentage for horse purslane at 30 DAE during 2019. It could be related to seed dispersal of horse purslane during previous season in the same field, which would have enriched soil seed bank and subsequent establishment of the weed during 2019. Moreover, it was observed that as the interference period progressed from 30 to 45 DAE, the frequency percentage increased in horse purslane-free and all weeds-free treatments until 20 DAE. This pattern is also understandable due to time advancement and progression in horse purslane life cycle and biology leading to peak vegetative growth at 45 DAE [17].

**Fig 6:** Frequency percentage of horse purslane at 30 (a) and 45 (b) days after emergence in soybean field. T_2_: Horse purslane-free till 20 DAE, T_5_: All weeds-free till 20 DAE, T_9_: Weedy check horse purslane only, T_10_: Weedy-check all weeds.

Different weed interference treatments significantly altered plant height of soybean during both years (Table 1). The highest plant height (67.22 and 73.43 cm) was recorded in all weeds-free treatment for whole season whereas weedy-check all weeds recorded the lowest plant height (39.48 and 44.39 cm) during 2018 and 2019. Increased plant height during second year could be due to the availability of abundant growth promoting factors in weed-free treatment that allowed soybean plants to attain their maximum height. No competition from weeds for sunlight and space in weed-free treatment would have resulted in expression of full genetic potential of crop plants. Plant height was reduced in weedy-check all weeds, including horse purslane treatment.

**Table 1:** The impact of interference of horse purslane and other weeds on plant height, number of pods plant^-1^ and 1000-grain weight of soybean during 2018 and 2019.

Treatments	Plant height (cm)		No. of pods plant^-1^	1000-grain weight (g)	
	2018	2019	Average over years	2018	2019
**T**_**1**_	67.22 a	73.43 a	80.70 a	104.24 a	107.19 a
**T**_**2**_	46.27 efg	49.61 g	57.31 ef	93.79 de	91.65 d
**T**_**3**_	50.45 cde	57.15 e	63.00 de	94.08 de	92.14 cd
**T**_**4**_	51.17 cd	61.91 c	65.00 cde	96.16 cd	97.50 b
**T**_**5**_	48.86 def	54.31 f	70.40c	92.56 ef	91.47 d
**T**_**6**_	54.58 bc	59.25 d	73.70 bc	98.41 bc	96.37 bc
**T**_**7**_	58.34 b	65.56 b	76.74 ab	100.36 b	103.49 a
**T**_**8**_	43.68 gh	47.39 h	62.96 de	88.75 g	89.09 d
**T**_**9**_	45.48 fg	49.41 g	65.50 cde	90.75 fg	87.71 d
**T**_**10**_	39.48 h	44.69 i	51.29 f	84.76 h	81.68 e
**Tukey’s HSD value**	4.219	0.568	6.230	2.514	4.617

**T**_**1**_: Weeds-free whole season, **T**_**2**_: Horse purslane-free till 20 DAE, **T**_**3**_: Horse purslane-free till 40 DAE, **T**_**4**_: Horse purslane-free till 60 DAE, **T**_**5**_: All weeds-free till 20 DAE, **T**_**6**_: All weeds-free till 40 DAE, **T**_**7**_: All weeds-free till 60 DAE, **T**_**8**_: All weeds-free except Horse purslane, **T**_**9**_: Weedy-check horse purslane only, **T**_**10**_: Weedy-check all weeds. Means sharing different letters differ significantly at 95% probability level.

The number of pods plant^-1^ were significantly altered by different treatments included in the study. However, year effect was non-significant; thus, mean data over years are presented (Table 1). Weed-free all weeds till 40 and 60 DAE recorded similar number of pods per plant. It suggests that probably 40 DAE are required for pods formation in soybean variety “Faisal soybean” used in this study. The lowest number of pods per plant were recorded in weedy-check all weeds treatment. The absence of weeds in weed-free treatment offered no competition to crop plants, thereby enhanced pod development and quantity [30].

Thousand-grain weight was significantly altered by weed interference treatments during both years (Table 1). The heaviest 1000-grains (104.24 g and 107.19 g) were recorded in weeds-free treatment for whole growing period, whereas the lightest 1000-grains (84.76 g and 81.68 g) were recorded in weedy-check all weeds treatment during 2018 and 2019. Weedy-check horse purslane only recorded the second lowest 1000-grain weight. This is quite possible as weed-free environment provide favorable conditions for the crop plants, which ultimately lead to better seed sink relationship and seed filling, resulting in heavier 1000 seeds. All weeds controlled until 60 DAE treatment also exhibited heavier 1000 seeds. Furthermore, all weeds-free for 40 DAE treatment also had almost similar weight of 1000 soybean seeds to all weeds-free for 60 DAE during both years. This trend is also similar to one obtained for number of pods per plant in the same treatment. It suggests that if weeds are kept out of soybean fields until 60 DAE then the photosynthates production, transport, accumulation and assimilation in economic part can be increased to higher level resulting in heavier seeds [17].

Seed yield was significantly influenced by different treatments during 2018 and 2109 (Table 2). The highest grain yield (1604.89, 2033.9 kg ha^-1^ during 1^st^ and 2^nd^ year, respectively) was recorded for weeds-free treatment during whole crop period. The lowest grain yield (980.48, 613.85 kg ha^-1^ during 1^st^ and 2^nd^ year, respectively) was recorded in weedy-check all weeds treatment. Soybean plots with weeds-free situation until 40 DAE or 60 DAE recorded statistically similar grain yield during both years of the study. Nonetheless, interference of horse purslane with weedy-check horse purslane only recorded the second lowest value for grain yield and harvest index. This indicates that horse purslane significantly altered yield and related traits. The presence of horse purslane alone resulted in significant yield reduction. Significant yield losses in soybean have also been attributed to horse purslane interference in earlier studies [31, 32]. There are negative allelopathic effects of horse purslane extracts on soybean productivity [33]. It indicates that horse purslane was more aggressive. The essential nutrients and resources would have been consumed more effectively by horse purslane.

**Table 2:** The impact of horse purslane and other weeds’ interference on grain yield and harvest index of soybean crop.

Treatments	Grain yield kg ha^-1^		Harvest index (%)	
	2018	2019	2018	2019
**T**_**1**_	1604.89 a	2033.90 a	24.55 a	30.26 a
**T**_**2**_	1166.27 e	963.88 ef	19.95 d	17.00 def
**T**_**3**_	1283.73 d	1045.38 de	21.05 c	17.86 cde
**T**_**4**_	1339.55 c	1415.80 bc	21.43 c	16.94 def
**T**_**5**_	1419.53 b	1193.78 cde	23.15 b	19.83 bcd
**T**_**6**_	1432.31 b	1360.74 bcd	22.84 b	23.83 b
**T**_**7**_	1449.56 b	1516.87 b	22.84 b	22.56 bc
**T**_**8**_	990.64 g	998.64 ef	18.55 e	18.26 cde
**T**_**9**_	1086.53 f	724.92 fg	19.81 d	13.75 ef
**T**_**10**_	980.48 g	613.85 g	19.17 de	12.48 f
**Tukey’s HSD value**	42.956	315.620	1.053	4.820

**T**_**1**_: Weeds-free whole season, **T**_**2**_: Horse purslane-free till 20 DAE, **T**_**3**_: Horse purslane-free till 40 DAE, **T**_**4**_: Horse purslane-free till 60 DAE, **T**_**5**_: All weeds-free till 20 DAE, **T**_**6**_: All weeds-free till 40 DAE, **T**_**7**_: All weeds-free till 60 DAE, **T**_**8**_: All weeds-free except Horse purslane, **T**_**9**_: Weedy-check horse purslane only, **T**_**10**_: Weedy-check all weeds. Means sharing different letters differ significantly at 95% probability level.

While comparing weedy-check plots with each other, it apparent that generally weedy-check all weeds treatment recorded the lowest grain yield. It depicts that the weeds infesting the area, i.e., false amaranth, purple nut sedge and horse purslane could have synergism to reduce soybean yield. Moreover, findings are evident of the fact that although horse purslane exerted heavy damage on soybean yield, the cumulative effect of all weeds in integration was more decisive regarding grain yield than the sole horse purslane. Akter et al. [33] also reported reduction in soybean yield due to weed competition. In the current study, soybean yield was reduced by 38.90 and 69.84% during 2018 and 2019, respectively by weedy-check all weeds treatment. Similarly, weedy-check horse purslane alone reduced soybean yield by 32.29 and 64.38% during 2018 and 2019. Soybean yield in weedy environment decreased by 36% compared with weed-free treatment [34].

The effect of different weed interference treatments on harvest index was significant during both the years. The highest harvest index (24.55 and 30.26% during 1^st^ and 2^nd^ year, respectively) was recorded for weeds-free whole season treatment. The lowest harvest index (19.17 and 12.48% during 1^st^ and 2^nd^ year, respectively) was recorded for weedy-check all weeds treatment. The significant increase in harvest index for weed-free treatments during the whole duration resulted in linked with higher grain yield as described above. The harvest index in weedy-check treatments reduced due to higher weed-crop competition and subsequent low yield [35].

Percent increase/decrease in grain yield by different weed interferences treatments was calculated as the treatments have significant effect (Fig 7). Significant increase in yield in weed-free whole season treatment was observed during both years. The yield was increased by 32.29 and 65.43% during 1^st^ and 2^nd^ year, respectively as no weed constraint was present that limited plant growth. It was noteworthy that plots where all weeds were allowed to grow for whole growing season reduced soybean yield over weedy-check horse purslane only. Weed-free whole season treatment was followed by plots where weeds were kept free until 60 DAE as their interval for critical crop competition was passed and less damage occurred to the crop. While comparing percent yield increase over the weedy-check horse purslane plots with horse purslane-free treatment until 40 DAE and all weeds-free until 40 DAE, it was noticed that yield was increased by 33.76 and 48.30%, respectively. Results showed that plots having all weeds during whole growing season reduced grain yield by 10% and 24% during 1^st^ and 2^nd^ year, respectively over weedy-check horse purslane only. Moreover, plots having all weeds except horse purslane during whole growing season also showed 10% decrease in grain yield during 2018. While in 2019, 28% increase in grain yield was recorded. Increased hors purslane interference and its uncontrolled growth and development negatively affected grain yield. Among three weedy-check treatments, yield reduction was weedy-check all weeds > weedy-check all weeds except horse purslane > weedy check horse purslane only.

**Fig 7:** Percentage increase in soybean yield over weedy-check horse purslane alone treatment.

During both years, horse purslane density stood 2^nd^, while looking at the accumulation of total dry matter, it produced more dry matter than other weeds present in the field. It showed that horse purslane used available resources more efficiently that other annual and perennial weeds. An increase in horse purslane infestation over the growing season from 2018 to 2019 was 21%. It is clear that horse purslane was most aggressive during 2019 that could be attributed to the environmental condition which supported its growth and development. As weeds found favorable condition, their growth and development is increased [36]. Horse purslane showed most aggressive growth and development until 6 weeks after emergence. Horse purslane growth and development was higher than other weeds. This indicates that to avoid the economic losses by horse purslane in summer grown soybean crop, it should be controlled efficiently until 40 DAE. These results are similar to the findings of Ugalechumi et al. [37] who revealed that higher horse purslane density can reduce growth and development of crop plants. Overall, weed infestation was higher at 30 DAE during both the growing years. Higher frequency percentage, relative frequency and density of horse purslane during 2019 is evident from Figs 4–6. These findings are supported by the results of Ara et al. [38] who stated that resource use efficiency of purple nut sedge was reasonably lower than horse purslane.

## Conclusion

If soybean fields are kept free form horse purslane until 40 DAE, it can increase grain yield by 15.36% yield as compared to horse purslane throughout the growing season. However, yield can be increased by 30% if all weeds are controlled until 40 DAE. Keeping field free from a single weed is not economically feasible. Horse purslane alone could not prove a single main cause of interference in soybean fields when compared with other prevalent weeds. If soybean fields are infested with more than two weeds, including horse purslane or heavily infested with horse purslane alone, farmers should control weeds during initial 40 DAE in either case for better soybean productivity.
